# LINC00174 Facilitates Cell Proliferation, Cell Migration and Tumor Growth of Osteosarcoma *via* Regulating the TGF-β/SMAD Signaling Pathway and Upregulating SSH2 Expression

This article has been retracted.

**DOI:** 10.3389/fmolb.2021.697773

**Published:** 2021-06-17

**Authors:** Changjun Zheng, Ronghang Li, Shuang Zheng, Hongjuan Fang, Meng Xu, Lei Zhong

**Affiliations:** ^1^ Department of Orthopedics, The Second Hospital of Jilin University, Changchun, China; ^2^ Department of Electric Diagnostic, The Fourth Hospital of Jilin University, Changchun, China

**Keywords:** OS, LINC00174, miR-378a-3p, SSH2, TGF-β/Smad

## Abstract

Osteosarcoma (OS), a frequent malignant tumor which mainly occurs in the bone. The roles of long noncoding RNAs (lncRNAs) have been revealed in cancers, including OS. LncRNA long intergenic non-protein coding RNA (LINC00174) has been validated as an oncogene in several cancers. However, the role of LINC00174 in OS has not been explored. In our research, loss-of-function assays were conducted to explore the function of LINC00174 in OS cells. Then, we explored the downstream pathway of LINC00174 in OS cells. Bioinformatics, RNA pull-down and RIP experiments investigated the downstream mechanism of LINC00174 in OS cells. Finally, *in vivo* assays clarified the effect of LINC00174 on tumorigenesis. We found that LINC00174 was upregulated in OS tissues and cells. LINC00174 knockdown repressed OS cell growth. Mechanistically, LINC00174 knockdown suppressed the TGF-β/SMAD pathway. LINC00174 interacted with miR-378a-3p, and slingshot protein phosphatase 2 (SSH2) 3′UTR was targeted by miR-378a-3p in OS cells. Rescue assays showed that SSH2 upregulation or miR-378a-3p inhibition counteracted the inhibitory effect of LINC00174 depletion in OS cell growth. Additionally, LINC00174 depletion suppressed tumor growth in mice. In conclusion, LINC00174 promotes OS cellular malignancy and tumorigenesis *via* the miR-378a-3p/SSH2 axis and the TGF-β/SMAD pathway, which might provide a novel insight for OS treatment.

## Introduction

Osteosarcoma (OS) is a common malignant tumor that develops in the bone and occurs most preferentially in adolescents and children (Dean et al., 2018). The most common location of OS is the long bone metaphysis and the commonest site is the distal femur, followed by the proximal tibia and humerus (Alfranca et al., 2015). To date, the therapies of OS including surgical excision accompanying with chemotherapy and radiotherapy were performed to prolong survival and ensure the optimum outcome (Hughes, 2009). Although great progress has been achieved in OS therapy, the survival time of patients with OS is still not optimistic (Luetke et al., 2014). Thus, investigating the underlying molecular mechanisms in OS is urgently needed for novel treatment in OS.

According to the transcript length, noncoding RNAs are divided into long noncoding RNAs (lncRNAs) (> 200 nucleotides) and small noncoding RNAs (< 200 nucleotides) (Yao et al., 2019). Emerging evidence has demonstrated that lncRNAs play vital roles in multiple tumor processes including cell proliferation, metastasis and apoptosis (Adams et al., 2017; Huo et al., 2017). Previous reports have represented that several lncRNAs were involved in OS progression. For example, downregulation of NCK-AS1 modulates cell resistance to cisplatin in OS (Cheng et al., 2019). LncRNA-CIR accelerates OS cell proliferation and represses cell apoptosis (Liu et al., 2019). Moreover, HIF-1α induced lncRNA FOXD2-AS1 could promote OS progression by repressing the expression of p21 (Ren et al., 2019). Recently, lncRNA long intergenic non-protein coding RNA (LINC00174) has been revealed to exert crucial roles in several cancers. LINC00174 promotes glioma cell proliferation, migration, invasion, and glycolysis and exerts a tumorigenesis role by promoting tumor growth *in vivo* (Shi et al., 2019). Another study has demonstrated that the upregulation of LINC00174 indicates the poor prognosis of colorectal cancer patients, and LINC00174 exerts an oncogenic role by facilitating colorectal cancer cell growth *in vitro* and tumor growth *in vivo* (Shen et al., 2018). Moreover, LINC00174 is upregulated in hepatocellular carcinoma tissues and promotes the malignant phenotypes of hepatocellular carcinoma cells (Zhao et al., 2020). However, its biological function in OS remains unclear.

MicroRNAs (miRNAs), another subgroup of ncRNAs, are approximately 22 nucleotides in length (Tutar, 2014). Emerging studies have revealed that miRNAs post-transcriptionally modulate expression of messenger RNAs (mRNA) by binding with the 3′untranslated region (3′UTR) of mRNAs in tumors (Nogales-Cadenas et al., 2016; Abreu et al., 2017). Furthermore, lncRNAs can bind to miRNAs as competing endogenous RNAs (ceRNAs), thereby affecting and regulating the expression of messenger RNAs (mRNAs) (Zhou et al., 2019). For instance, lncRNA XIST regulates the miR-137/EZH2 axis to promote tumor metastasis in colorectal cancer (Liu et al., 2018). Additionally, PVT1 promotes tumor progression by regulating the miR-143/HK2 axis in gallbladder cancer (Chen et al., 2019). We intended to investigate whether there is such regulatory mechanism mediated by LINC00174 in OS progression.

In our present study, we aimed to probe the biological role and molecular mechanism of LINC00174 in OS progression. Our research may provide a potential novel insight for the therapeutic strategies of OS.

## Materials and Methods

### Tissue Samples

A total of 42 paired OS samples and adjacent normal tissues were obtained from OS patients who had not received chemotherapy or radiotherapy before surgery at the Second Hospital of Jilin University (Jilin, China). The patients all signed informed consents. These collected tissues were maintained at −80°C after surgery resection. The research was performed with the approval of the Ethics Committee of the Second Hospital of Jilin University (Jilin, China).

### Cell Culture and Transfection

Normal human osteoblast cell line (NHost) and OS cell lines (KHOS, U2OS, and MG63) were obtained from Cell Bank of the Chinese Academy of Sciences (Shanghai, China). Cells were incubated in Dulbecco’s Modified Eagle’s Medium (DMEM; Gibco, United States) containing 10% fetal bovine serum (FBS; Gibco, United States) and 1% penicillin/streptomycin (Invitrogen, United States) in a humid atmosphere with 5% CO_2_ at 37°C.

MG63 and U2OS cells were plated into 96-well plates (2 × 10^4^cells/well). Short hairpin RNA (shRNA; 20–50 nM) targeting LINC00174 (sh-LINC00174) and its negative control (sh-NC), miR-378a-3p inhibitor or miR-378a-3p mimics) and their controls (20–50 nM), and 1 μg of pcDNA3.1-slingshot protein phosphatase 2 (SSH2) vectors were obtained from Genepharma (Shanghai, China). Cell transfection was conducted using Lipofectamine 3,000 reagent (Invitrogen, United States) under manufacturer’s instructions. After 48 h of transfection, cells were then collected for the following assays.

To obtain stably LINC00174-downregulated OS cells, sh-NC and the sh-LINC00174 were transfected into MG63 cells with a lentivirus, then stable cells were selected with puromycin.

### RNA Extraction and Reverse Transcription Quantitative Real-Time Polymerase Chain Reaction

Total RNA was extracted from cultured cells or human tissues or mouse tissues by TRIzol reagent (Invitrogen, Shanghai, China) strictly following the instructions. Reverse transcription for LINC00174 was performed with PrimeScript RT Master Mix (Takara Bio, Inc., Dalian, China). Reverse transcription for mRNAs was performed from total RNA using a High Capacity cDNA Reverse Transcription (ThermoFisher) kit under the manufacturer’s instruction. Synthesis of complementary DNA (cDNA) was performed using the TaqMan® MicroRNA Reverse Transcription (Applied Biosystems) kit containing primers for miR-150-5p and miR-378a-3p that were obtained from the TaqMan® MicroRNA Assays (ThermoFisher) under the manufacturer’s instructions. Gene expression of LINC00174 and mRNAs was quantified by real-time PCR using Fast Real-Time PCR System (Applied Biosystems). PCR reactions for miRNAs were performed using TaqMan Universal Master Mix (Applied Biosystems) containing oligonucleotides and probes TaqMan® MicroRNA Assay (Applied Biosystems). Glyceraldehyde-3-phosphate dehydrogenase (GAPDH) and RNU6 (U6) act as internal controls for lncRNA (or mRNAs) and miRNAs, respectively. The 2^−ΔΔCt^ method was used to calculate relative expression levels of genes. The sequences of primers used in this research were shown in Supplementary Table S1.

### Cell Counting Kit 8 Assay

CCK-8 (Dojindo, Japan) was performed to test OS cell proliferation. In brief, MG63 and U2OS cells were placed in 96-well plates (2 × 10^4^/well). CCK-8 solution was supplemented after transfection for 0, 24, 48, and 72 h. After 4 h of incubation, the optimal density (OD) value at 450 nm was detected using a Bio-Rad 3,550 microplate reader (Bio-Rad, United States).

### Colony Formation Assay

Briefly, transfected MG63 and U2OS cells were plated in 6-well plates with approximately 1 × 10^3^ cells per well and cultured at 37°C for 14 days until colonies are visible. Colonies were then immobilized by methanol and dyed by 0.1% crystal violet. The number of colonies containing over 50 cells were manually counted.

### Wound Healing Assay

Wound healing assay was used to detect the OS cell migration ability. Briefly, MG63 and U2OS cells were placed in 6-well plates (1 × 10^4^ cells/well) and allowed to reach confluence. After scratching with a pipette tip, cells were cultured at 37°C for 24 h. The relative wound width was detected, photographed at 0 and 24 h through Olympus microscopy (Olympus, Japan) after scratching. The migration ability was evaluated by ImageJ software (National Institutes of Health, United States).

### Transwell Assays

The migratory and invasive abilities of OS cells were evaluated by Transwell assays with the Transwell chamber (Corning, United States). Transfected MG63 and U2OS cells were suspended in DMEM with 10% FBS in the bottom chamber and then 200 μL of cell suspension containing 1 × 10^5^ cells were put into the upper chamber with the membrane coated with (for the cell invasion assay) or without (for the cell migration assay) Matrigel (Thermo Fisher Scientific, United States). After two days, the migrated or invaded cells were fixed in methanol and then stained with 0.5% crystal violet. Finally, the migrated or invaded cells were observed and counted by Olympus microscopy (Olympus, Japan).

### Western Blot

Total protein was isolated from OS cells and xenograft tumor tissues by Radio Immunoprecipitation Assay lysis buffer. After separating by 10% sodium dodecyl sulfate polyacrylamide gel, proteins were then moved to polyvinylidene fluoride membranes (Millipore, United States). Then, the membranes were blocked with 5% nonfat milk, incubated with primary antibodies against GAPDH (ab181602, 1:10,000; Abcam, Shanghai, China), transforming growth factor-β1 (TGF-β1; ab179695, 1:1,000), SMAD2 (ab33875, 1:1,000), SMAD3 (ab40854, 1:1,000), Smad2 (phospho S255) (ab188334, 1:2,000), Smad2 (phospho S467) (ab53100, 1:500), Smad3 (phospho T179) (ab193297, 1:1,000), Smad3 (phospho S213) (ab63403, 1:1,000), Smad3 (phospho S423/S425) (ab52903, 1:2,000), and Ki67 (ab16667, 1:1,000) at 4°C overnight, followed by incubation with secondary antibody for 1 h at darkness. The relative levels of proteins were evaluated using an ECL chemiluminescent detection system (Thermo Fisher Scientific, Rochester. NY).

### RNA Pull-Down Assay

Biotinylated LINC00174 (LINC00174 probe-biotin) and negative control (LINC00174 probe-no biotin) purchased from Sangon (Shanghai, China) were transfected into MG63 and U2OS cells. The cells were lysed and collected after transfection. After incubation with Dynabeads M-280 Streptavidin (Invitrogen) for 10 min, the bound RNAs were subjected to RT-qPCR for quantification and analysis.

### Dual Luciferase Reporter Assay

The binding site between miR-378a-3p and LINC00174 (or SSH2 3′UTR) was predicted through starBase v2.0 (http://starbase.sysu.edu.cn/). The pGL3 luciferase reporters (Promega, Madison, WI) constructed with wild-type (Wt) or mutant (Mut) sequences of LINC00174 or SSH2 3′UTR were generated. Then, the constructed Wt (or Mut) luciferase reporters were co-transfected with miR-378a-3p mimics (or NC mimics) in MG63 and U2OS cells by Lipofectamine 2,000 reagent (Invitrogen, United States). After 48 h of transfection, the relative luciferase activities were analyzed using a dual-luciferase reporter assay system (Promega, United States).

### RNA Immunoprecipitation Assay

RIP assay was performed using an EZ-Magna RIP Kit (Millipore, United States). In brief, MG63 and U2OS cells were lysed in complete RIP lysis buffer, and then whole cell extract (100 µL) was incubated with magnetic beads conjugated with Ago2 or normal IgG antibody. All antibodies were obtained from Abcam (Shanghai, China). After washing the beads, the complexes were treated with the Proteinase K to remove proteins. Finally, the expression of LINC00174 and miR-378a-3p were detected through RT-qPCR.

### Subcellular Fractionation Assay

This assay was operated using a PARIS Kit (Life Technologies, United States) under the supplier’s instructions. After the nuclear and cytoplasmic fractions of MG63 and U2OS cells were separated, the expression of LINC00174 and miR-378a-3p was measured by RT-qPCR with GAPDH and U6 as cytoplasmatic and nuclear internal controls, respectively.

### Ethics Statement

In this study, animal management was performed strictly in line with the Guide for the Care and Use of Laboratory Animals by the National Research Council Institute (United States) for Laboratory Animal Research. Animal experiments were approved by the Ethics Committee of The Second Hospital of Jilin University (Jilin, China).

### Tumor Xenograft Assays

BALB/c nude mice (4-week-old, Vital River, Beijing, China; *n* = 3 mice/group) were obtained. For tumorigenesis assays, stably transfected MG63 cells (5 × 10^6^ cells/mL) with lentivirus carrying sh-LINC00174 or sh-NC were subcutaneously injected into the mice. Tumor growth was tested and recorded every 7 days. Tumor volume was calculated (equation V (volume) = L (longitudinal diameter) × W (latitudinal diameter) ^2^/2). After one month, the mice were sacrificed, and then the xenograft tumors in each mouse were resected, photographed, and weighed. The tumor tissues were stored at −80°C for following RT-qPCR and western blot analysis.

### Statistical Analysis

All experiments were performed in triplicate and the data were represented as mean ± standard deviation. SPSS 19.0 (IBM, United States) was used for statistical analyses. Student’s *t* test was performed to compare the differences between two groups. One-way analysis of variance with Tukey’s *post hoc* test was used to measure differences of multiples groups. *p* < 0.05 was regarded statistically significant.

## Results

### LncRNA LINC00174 Is Upregulated in OS Tissues and Cells

LINC00174 was reported to be upregulated and serve as an oncogene in glioma cells (Shi et al., 2019). Its role in OS remains elusive. First, LINC00174 expression status in 42 OS tissue samples and the paired adjacent normal tissues was measured. RT-qPCR results revealed that LINC00174 was upregulated in OS tissues compared to in adjacent normal tissues (Figure 1A). Next, we detected LINC00174 expression in OS cell lines (KHOS, MG63, and U2OS) and normal osteoblastic cell line NHost. As shown in Figure 1B, LINC00174 expression was upregulated in OS cells, particularly much higher in MG63 and U2OS cells.

**FIGURE 1:** LncRNA LINC00174 is upregulated in OS tissues and cell lines. **(A)** The expression of LINC00174 in 42 OS tissue samples and matched adjacent normal tissues was measured by RT-qPCR. *n* = 42. Significance was analyzed by Student’s t-test. **(B)** The expression of LINC00174 in OS cell lines (KHOS, MG63, and U2OS cells) and the normal osteoblastic cell-line NHost was detected by RT-qPCR. Significance was analyzed by Student’s t-test. *p < 0.05.

### LINC00174 Silencing Suppresses OS Cell Proliferation, Migration and Invasion

To probe the biological function of LINC00174 in OS cells, the loss-of-function assays were performed in MG63 and U2OS cells. First, the knockdown efficacy of LINC00174 was measured by RT-qPCR. The results suggested that LINC00174 expression in MG63 and U2OS was decreased under transfection with sh-LINC00174 (Figure 2A). Next, the viability of MG63 and U2OS cells was measured by CCK-8 assay. We found that OS cell viability was inhibited under LINC00174 knockdown (Figure 2B). Additionally, the results of colony formation assay revealed the decreased number of colonies in MG63 and U2OS cells transfected with sh-LINC00174 (Figures 2C,D). Wound healing and Transwell assays demonstrated that the invasion and migration of OS cells were suppressed under downregulation of LINC00174 (Figures 2E–G).

**FIGURE 2:** LINC00174 knockdown inhibits OS cell proliferation, migration and invasion. **(A)** The transfection efficacy of sh-LINC00174 or sh-NC in U2OS and MG63 cells was examined by RT-qPCR analysis. Significance was analyzed by Student’s t-test. **(B)** CCK-8 assay was used to evaluate the viability of U2OS and MG63 cells transfected with sh-LINC00174 and sh-NC. Significance was analyzed by Student’s t-test. **(C,D)** Colony formation assay was used to measure the proliferation of U2OS and MG63 cells transfected with sh-LINC00174 and sh-NC. Significance was analyzed by Student’s t-test. **(E)** Wound healing assay was used to determine the migration of OS cells transfected with sh-LINC00174 and sh-NC. Significance was analyzed by Student’s t-test. **(F,G)** Transwell assays were used to detect the migration and invasion of OS cells transfected with sh-LINC00174 and sh-NC. Significance was analyzed by Student’s t-test. *p < 0.05.

### LINC00174 Knockdown Inhibits the TGF-β/SMAD Pathway

The TGF-β/SMAD signaling pathway has been revealed to participate in OS development, and is activated in OS cells (Johnsen et al., 2002; Lamora et al., 2014). TAZ, a transcriptional coactivator with PDZ-binding motif, is encoded by WW domain containing transcription regulator one gene (WWTR1). TAZ is tightly regulated in the hippo pathway-dependent and -independent manner in response to a wide range of extracellular and intrinsic signals (Zhou and Lei, 2016; Totaro et al., 2018). LINC00174 has been reported to facilitate colorectal carcinoma progression through regulating TAZ (Shen et al., 2018). Moreover, TAZ/YAP dictates the localization of active SMAD complexes in response to cell density-mediated formation of polarity complexes. In high-density cell cultures, the Hippo pathway drives cytoplasmic localization of TAZ/YAP, which sequesters SMAD complexes, thereby suppressing TGF-β signaling (Varelas et al., 2010). Accumulating studies have verified that TAZ retains SMAD complexes on DNA, and then regulates the TGF-β/SMAD signaling pathway (Szeto et al., 2016; Pagiatakis et al., 2017; Qin et al., 2018). Thus, we wondered whether LINC00174 can regulate the TGF-β/SMAD pathway in OS. RT-qPCR analysis validated the reduced mRNA expression levels of TGF-β1, SMAD2 and SMAD3 in both MG63 and U2OS cells under depletion of LINC00174 (Figure 3A). Subsequently, western blot analysis verified the decreased protein levels of TGF-β1, SMAD2, and SMAD3 in OS cells under LINC00174 silencing (Figure 3B). Moreover, we detected expression of Smad2 (phospho S255), Smad2 (phospho S467), Smad3 (phospho T179), Smad3 (phospho S213), Smad3 (phospho S423/S425) proteins in MG63 and U2OS cells in the presence and absence of LINC00174. The results showed that phosphorylated Smad2 (S255) protein and phosphorylated Smad3 (T179) protein showed significant downregulation in cells transfected with sh-LINC00174 compared to that in cells transfected with sh-NC (Figure 3C).

**FIGURE 3:** LINC00174 knockdown inhibits the TGF-β/SMAD pathway. **(A)** The mRNA expression levels of TGF-β1, SMAD2, and SMAD3 in OS cells in sh-LINC00174 or sh-NC group was determined by RT-qPCR analysis. Significance was analyzed by Student’s t-test. **(B)** Western blot was performed to measure the protein levels of TGF-β1, SMAD2, and SMAD3 in OS cells in sh-LINC00174 or sh-NC group. Significance was analyzed by Student’s t-test. **(C)** Expression of Smad2 (phospho S255), Smad2 (phospho S467), Smad3 (phospho T179), Smad3 (phospho S213), Smad3 (phospho S423/S425) in MG63 and U2OS cells in the presence and absence of LINC00174 was detected by western blotting. Significance was analyzed by Student’s t-test. *p < 0.05.

### LINC00174 is a Molecular Sponge for miR-378a-3p

LncRNAs have been revealed to exert regulation in numerous human cancers as ceRNAs (Karreth and Pandolfi, 2013; Wang et al., 2019). Additionally, LINC00174 has been reported to competitively bind with miRNAs to modulate target gene expression in glioma and hepatocellular carcinoma progression (Shi et al., 2019; Zhao et al., 2020). We hypothesized that LINC00174 may exert its regulatory function on OS cellular behaviors in such manner. Thus, the downstream miRNAs of LINC00174 in OS cells were explored. First, the potential candidate miRNAs which might bind with LINC00174 were predicted by starBase database. MiR-150-5p and miR-378a-3p were obtained with the following conditions: high stringency in CLIP data (≥3); Pan-cancer ≥ 6 cancer types. Moreover, RNA pull-down assay results demonstrated that miR-378a-3p presented a significant enrichment and miR-150-5p showed no enrichment in complexes pulled down by biotinylated LINC00174 in OS cells (Figure 4A). Therefore, we selected miR-378a-3p for further study. RT-qPCR analysis suggested that overexpression of miR-378a-3p decreased LINC00174 level, and miR-378a-3p inhibitor increased LINC00174 expression in OS cells (Figure 4B). The binding fragment of miR-378a-3p on LINC00174 was predicted by starBase (Figure 4C). Then luciferase reporter assay was performed to clarify the binding of LINC00174 and miR-378a-3p. MiR-378a-3p mimics reduced the luciferase activity of LINC00174-Wt reporters in OS cells and the luciferase activity of LINC00174-Mut reporters in OS cells had no significant change (Figure 4D). These data verified that miR-378a-3p negatively affected the transcript stability of LINC00174 in OS cells. In addition, the corresponding schematic explained the major constituents of this luciferase reporter assay (Figure 4E). As shown in Figure 4F, both miR-378a-3p and LINC00174 were enriched in magnetic beads coated with anti-Ago2, indicating the interaction of LINC00174 and miR-378a-3p in OS cells. Furthermore, subcellular fractionation assay confirmed the cytoplasmatic colocalization of LINC00174 and miR-378a-3p in MG63 and U2OS cells (Figure 4G), suggesting that LINC00174 served as a miR-378a-3p sponge in OS cells. Moreover, miR-378a-3p expression was downregulated in OS tissues compared to that in adjacent nontumor tissues (Figure 4H).

**FIGURE 4:** LINC00174 is a molecular sponge for miR-378a-3p. **(A)** RNA pull-down assay was used to measure the enrichment of predicted miRNAs in pellets pulled down by biotinylated LINC00174 in OS cells. Significance was analyzed by Student’s t-test. **(B)** The expression of LINC00174 in OS cells in NC mimics, miR-378a-3p mimics, NC inhibitor or miR-378a-3p inhibitor group was detected by RT-qPCR. Significance was analyzed by Student’s t-test. **(C)** The predicted binding site between LINC00174 and miR-378a-3p was obtained from starBase. **(D)** Luciferase reporter assay assessed the binding ability between LINC00174 and miR-378a-3p in OS cells. Significance was analyzed by Student’s t-test. **(E)** Corresponding schematic diagram of luciferase reporter plasmid. **(F)** RIP assay was used to evaluate the binding ability between LINC00174 and miR-378a-3p in OS cells. Significance was analyzed by Student’s t-test. **(G)** Subcellular fractionation assay detected the colocalization of LINC00174 and miR-378a-3p in OS cells. **(H)** MiR-378a-3p expression in OS tissues and adjacent nontumor tissues was detected by RT-qPCR. Significance was analyzed by Student’s t-test. *p < 0.05, **p < 0.01.

### MiR-378a-3p Upregulation Suppresses the TGF-β/SMAD Pathway

The function of miR-378a-3p on the TGF-β/SMAD pathway was further explored. RT-qPCR analysis depicted that mRNA levels of TGF-β1, SMAD2, and SMAD3 in MG63 and U2OS cells were reduced under miR-378a-3p overexpression (Figure 5A). Furthermore, western blot results illustrated that miR-378a-3p mimics reduced the protein levels of TGF-β1, SMAD2, *p*-SMAD2 (S255), SMAD3, and *p*-SMAD3 (T179) in OS cells (Figures 5B,C).

**FIGURE 5:** MiR-378a-3p upregulation suppresses the TGF-β/SMAD pathway. **(A)** The mRNA expression levels of TGF-β1, SMAD2 and SMAD3 in OS cells transfected with NC mimics or miR-378a-3p mimics were determined by RT-qPCR analysis. Significance was analyzed by Student’s t-test. **(B,C)** Western blot measured the protein levels of TGF-β1, SMAD2, SMAD2 (phospho S255), SMAD3, and SMAD3 (phospho T179) in OS cells transfected with sh-LINC00174 or sh-NC group. Significance was analyzed by Student’s t-test. *p < 0.05.

### SSH2 is the Target Gene of miR-378a-3p

To further investigate the LINC00174-mediated ceRNA network, we searched the targets of miR-378a-3p in OS cells. Two candidate mRNAs (SSH2 and WRB) were found from starBase (condition: high stringency ≥ 3 on degradome data), with the overlapped results of PITA, microT and miRanda databases (Figure 6A). We then tested the expression levels of these two genes through RT-qPCR analysis. The results suggested that SSH2 mRNA level in OS cells was reduced by miR-378a-3p upregulation and increased by miR-378a-3p downregulation, and WRB mRNA level in OS cells showed no significant change under miR-378a-3p overexpression or depletion (Figures 6B–D). Subsequently, we measured the expression of SSH2 in OS cells by RT-qPCR analysis. We found that SSH2 expression was upregulated in OS cell lines compared to that in normal control cells (Figure 6E). Additionally, RT-qPCR results showed that SSH2 level was higher in OS tissues than in adjacent normal tissues (Figure 6F). As presented in Figure 6G, the potential binding site between miR-378a-3p and SSH2 3′UTR was predicted through starBase v2.0. Luciferase reporter assay results indicated that miR-378a-3p mimics reduced the luciferase activity of SSH2 3′UTR-Wt reporters rather than SSH2 3′UTR-Mut reporters in OS cells (Figure 6H). Furthermore, western blot suggested that SSH2 protein level was reduced in response to miR-378a-3p overexpression (Figure 6I).

**FIGURE 6:** SSH2 is the target gene of miR-378a-3p. **(A)** The potential mRNAs of miR-378a-3p from PITA, microT and miRanda under the condition of high stringency ≥ 3 on degradome data. **(B)** The expression of SSH2 or WRB in OS cells in NC mimics or miR-378a-3p mimics group was tested by RT-qPCR. Significance was analyzed by Student’s t-test. **(C,D)** The expression of SSH2 or WRB in OS cells transfected with NC inhibitor or miR-378a-3p inhibitor was examined by RT-qPCR. Significance was analyzed by Student’s t-test. **(E)** The expression of SSH2 in OS cell lines and the normal NHost cells was detected by RT-qPCR analysis. Significance was analyzed by Student’s t-test. **(F)** The expression of SSH2 in OS tissues and matched normal tissues was detected by RT-qPCR analysis. *n* = 42. Significance was analyzed by Student’s t-test. **(G)** The binding site between miR-378a-3p and SSH2 3′UTR. **(H)** The luciferase reporter assay was used to verify the binding ability between miR-378a-3p and SSH2 in OS cells. Significance was analyzed by Student’s t-test. **(I)** Western blot measured SSH2 protein level in OS cells transfected with NC mimics or miR-378a-3p mimics. Significance was analyzed by Student’s t-test. *p < 0.05.

### LINC00174 Aggravates OS Cellular Malignancy and Activates the TGF-β/SMAD Pathway *via* Modulating the miR-378a-3p/SSH2 Axis

To further clarify whether the miR-378-3p/SSH2 axis is involved in the LINC00174-mediated OS cellular processes, we performed the following rescue assays. First, OS cell viability and proliferation inhibited by sh-LINC00174 were reversed under SSH2 upregulation or miR-378a-3p downregulation (Figures 7A,B). Moreover, the decreased OS cell migration and invasion under LINC00174 silencing were rescued by SSH2 overexpression or miR-378a-3p depletion (Figures 7C,D). Furthermore, we found that SSH2 upregulation or miR-378a-3p deficiency counteracted the inhibitory effect of LINC00174 silencing on the TGF-β/SMAD pathway-related protein levels (Figure 7E).

**FIGURE 7:** LINC00174 promotes cell proliferation, migration and invasion and activates the TGF-β/SMAD pathway in OS progression by regulating the miR-378a-3p/SSH2 axis. **(A,B)** Cell viability and proliferation in MG63 cells in each group was detected using CCK-8 and colony formation assays. Significance was analyzed by ANOVA followed by Tukey’s *post hoc* test. **(C,D)** The migration and invasion of OS cells by different transfection conditions were measured by wound healing and Transwell assays. Significance was analyzed by ANOVA followed by Tukey’s *post hoc* test. **(E)** The protein levels of TGF-β1, SMAD2, SMAD2 (phospho S255), SMAD3, and SMAD3 (phospho T179) in MG63 cells in each group were evaluated by western blot analysis. Significance was analyzed by ANOVA followed by Tukey’s *post hoc* test. *p < 0.05.

### LINC00174 Facilitates OS Tumor Growth *in vivo*

Above findings suggested that LINC00174 promoted OS cell malignancy. We intended to further explore the role of LINC00174 in OS tumorigenesis. Therefore, we investigated the function of LINC00174 *in vivo* through xenograft tumor experiments. MG63 cells infected with lentivirus expressing sh-LINC00174 or sh-NC were subcutaneously injected into the mice. No visible tumor focus was found in lungs and livers of the xenograft nude mice. As shown in Figure 8A, LINC00174 knockdown significantly decreased the tumor volume. Moreover, LINC00174 silencing reduced the tumor size and weight (Figure 8B). Additionally, western blot analysis depicted that the level of Ki67 was declined in xenograft tumor tissues under LINC00174 downregulation (Figure 8C). Additionally, RT-qPCR analysis demonstrated that the expression levels of LINC00174 and SSH2 in xenograft tumor tissues were downregulated, and miR-378a-3p expression in xenograft tumor tissues was elevated under LINC00174 knockdown (Figure 8D). Western blot analysis suggested that LINC00174 deficiency reduced SSH2 protein level in xenograft tumor tissues (Figure 8E). Moreover, the TGF-β1 signaling pathway was inhibited in tumors of mice after treatment with MG63 cells infected with lentivirus expressing sh-LINC00174, as evidenced by the decreased TGF-β1, SMAD2, *p*-SMAD2 (S255), SMAD3, and *p*-SMAD3 (T179) protein levels (Figure 8F).

**FIGURE 8:** LINC00174 promotes OS progression *in vivo*. **(A)** The tumor volume was recorded under LINC00174 knockdown. *n* = 3. Significance was analyzed by Student’s t-test. **(B)** Tumor images and tumor weight under LINC00174 silencing. *n* = 3. Significance was analyzed by Student’s t-test. **(C)** The expression of Ki67 in xenograft tumor tissues in each group was determined by western blot. *n* = 3. **(D)** Expression levels of LINC00174, miR-378a-3p and SSH2 in xenograft tumor tissues were examined by RT-qPCR. *n* = 3. Significance was analyzed by Student’s t-test. **(E)** SSH2 protein level in xenograft tumor tissues under LINC00174 deficiency was measured by western blot. *n* = 3. Significance was analyzed by Student’s t-test. **(F)** TGF-β1, SMAD2, SMAD2 (phospho S255), SMAD3, and SMAD3 (phospho T179) protein levels in xenograft tumor tissues under LINC00174 deficiency was measured by western blot. *n* = 3. Significance was analyzed by Student’s t-test. *p < 0.05.

## Discussion

LINC00174 has been reported to act as an oncogene in glioma and hepatocellular carcinoma progression (Shi et al., 2019; Zhao et al., 2020). In this work, the upregulated expression of LINC00174 was verified in OS tissues and cells. Moreover, downregulation of LINC00174 suppressed cell proliferation, migration, and invasion in OS cells. In addition, LINC00174 depletion repressed OS tumor growth *in vivo*. Our findings implied that LINC00174 served as an oncogene in OS progression by promoting cell malignancy *in vitro* and tumorigenesis *in vivo*.

TGF-β has been revealed to regulate tumor cellular behaviors, such as cell proliferation, cell growth and cell migration (Jung et al., 2017; Batlle and Massagué, 2019). Furthermore, TGF-β activates several biological pathways, including the SMAD2 (García-Vizcaíno et al., 2017), SMAD3 (Ooshima et al., 2019) and PI3K/Akt (Li et al., 2019) pathways. Furthermore, accumulating evidence has demonstrated that the TGF-β/SMAD pathway is involved in OS progression. For instance, miR-522 promotes osteosarcoma tumorigenesis by targeting PPM1A via the TGF-β/SMAD signaling pathway (Xu and Liu, 2019). In addition, GDF15 promotes osteosarcoma cell migration and invasion by regulating the TGF-β signaling pathway (Chen et al., 2019). In this work, we found that LINC00174 knockdown inactivated the TGF-β/SMAD pathway in OS cells by inhibiting the phosphorylation of Smad2 at S255 and by inhibiting the phosphorylation of Smad3 at T179. These findings suggested that LINC00174 promoted cell malignancy and tumorigenesis *via* activation of the TGF-β/SMAD pathway.

LncRNAs, serve as ceRNAs, can abrogate the endogenous effect of miRNAs on their target mRNAs (Karreth and Pandolfi, 2013; Wang et al., 2019). It has been previously reported that the ceRNA regulatory network of lncRNA/miRNA/mRNA exerts vital effect on carcinogenesis of many tumors (Bai et al., 2019; Luan et al., 2020; Ma et al., 2020). MiR-378a-3p has been revealed to exert as a tumor suppressor in some cancers. For instance, miR-378a-3p suppresses ovarian cancer cell proliferation and promotes sensitivity of ovarian cancer cells to cisplatin (Xu et al., 2018). Another report has demonstrated that miR-378a-3p inhibits the viability, proliferation, migration and invasion of the esophageal squamous cell carcinoma cells (Ding et al., 2018). Moreover, miR-378a-3p represses cellular proliferation and migration in glioblastoma multiforme (Guo et al., 2019). In this work, we used bioinformatics to explore the potential miRNAs binding with LINC00174. MiR-378a-3p was found as putative downstream molecule of LINC00174. Mechanistically, miR-378a-3p bound with LINC00174 in OS cells. MiR-378a-3p negatively modulated LINC00174 expression. Furthermore, we found the cytoplasmatic colocalization of LINC00174 and miR-378a-3p in OS cells. These findings suggested that LINC00174 served as a miR-378a-3p sponge in OS cells. Additionally, miR-378a-3p exerted a suppressive effect on the TGF-β/SMAD pathway in OS cells.

SSH2 belongs to a gene family composed of three members (SSH1, SSH2, and SSH3) that have been revealed to modulate essential cellular processes, including migration and invasion. SSH2 family members are required for the effective migration and invasion of tumor cells through maintenance of the unidirectionality of membrane protrusions (Niwa et al., 2002). SSH2 was reported to be upregulated in colorectal cancer cells and promote proliferation of colorectal cancer stem cells (Sun et al., 2019). In our research, SSH2 was predicted as a candidate target of miR-378a-3p. We found that SSH2 was upregulated in OS tissues and cells. Mechanical experiments verified that miR-378a-3p targeted SSH2 3′UTR and reduced SSH2 mRNA and protein levels. Through rescue experiments, we found that SSH2 upregulation or miR-378a-3p downregulation rescued the decreased OS cell proliferation, migration, invasion and the inactive TGF-β/SMAD signaling under LINC00174 silencing. These findings suggested that LINC00174 mediated OS cellular processes and the TGF-β/SMAD signaling through sponging miR-378a-3p and regulating SSH2 expression.

In conclusion, the current research revealed that the LINC00174/miR-378a-3p/SSH2 axis facilitated cellular malignancy and tumor growth via the TGF-β/SMAD signaling pathway in OS progression. This discovery might provide a novel insight for the further exploration of OS treatment. However, there are some limitations in the design of our research. Current attempt only identified Ago2 crosslinks that are even more common in 5′UTRs and CDS compared to 3′UTR, indicating that not every Ago2 crosslink cluster represents a bona fide miRNA target site. Therefore, it is required to support the proposed sponging mechanism with alternative orthogonal experiment. Additionally, a fascinating cross-talk with TGF-β signaling, remains unexplained.

## Data Availability

The original contributions presented in the study are included in the article/Supplementary Material, further inquiries can be directed to the corresponding author.
